This article has been retracted.

# Research on Cancer Molecular Typing Based on High-Throughput Sequencing Technology

**DOI:** 10.1155/2021/9941475

**Published:** 2021-12-07

**Authors:** Dan Wei

**Affiliations:** ^1^Department of Laboratory Medicine, The Third Xiangya Hospital of Central South University, Changsha City, Hunan Province, China 410013; ^2^Department of Laboratory Medicine, Xiangya Medical School, Central South University, Changsha City, Hunan Province, China 410013

## Abstract

This paper studies the role of high-throughput measurement technology in cancer molecular typing. Based on the Dendrix algorithm, the model proposed in this paper selects the gene replication time as an inherent attribute that affects the frequency of gene mutations and adds it to the model. After setting the size of the gene set, compared with the Dendrix algorithm, the model does not need to delete the gene set that has been found in the process of searching the pathway, and it can find more driving pathway gene sets. Based on the high coverage and high exclusivity of the driving gene set in the pathway and the influence of gene covariates, this paper constructs an adaptive multiobjective optimization model. In order to overcome the problem of gene mutation heterogeneity, this model introduces gene covariates as the weight of gene mutation frequency so that the model is adaptive to each gene. The analysis of the research results shows the reliability of high-throughput sequencing technology.

## 1. Introduction

With the rapid development and promotion of high-throughput sequencing technology, many international scientific research institutions have hosted large-scale cancer genome sequencing projects. With the maturity of sequencing technology for large-scale samples, cancer researchers have shifted their focus to mining based on cancer big data. A large amount of biological data has laid a solid foundation for researchers to re-understand cancer. Since the 21st century, research on data mining and identification based on cancer data has sprung up. In a cancer review study, Professor Weinberg briefly described recent hotspots and progress in oncology and proposed some professional concepts in malignant tumors, including tumor cell characteristics, autophagy, tumor microenvironment, and tumor stem cells [1]. These studies have far-reaching significance for revealing the pathogenesis of cancer.

Although cancer's high death rate is concerning, human knowledge of cancer is woefully inadequate at this point. Few people understand the underlying issues that lead to malignant tumors, including what causes tumors to begin with and what causes them to spread and proliferate once they have metastasized. These questions and others like them must be addressed immediately. Except for a few diseases, the 40-year “war against cancer” has been a failure. [2]. Early detection and therapy may be utilized to reduce tumor mortality or considerably prolong the lives of tumor patients, thanks to the fast advancement of contemporary medical technology. However, relying simply on early prevention is insufficient if you want to thoroughly win the ultimate victory in the war against malignant tumors. By incorporating molecular and genetic feature information into the categorization system, more relevant prognostic information may be obtained, and the impacts of new medications can be predicted. [3]. At present, great efforts have been made to explore new molecular markers, among which gene expression profiling has been proven to be an effective method that can be used to group tumors and predict the prognosis of cancer patients [4]. Many novel molecular markers have recently been found, and they have been shown to help speed up diagnosis and improve outcomes for women with endometrial cancer. Gene expression profile data or protein chips have also been used to identify certain molecular markers, and a prognosis model has been developed [5]. These known prognostic indicators are challenging to utilise in clinical practice since they only apply to partial staging and/or tissue grade of endometrial cancer. A predictive model with high resolution capabilities is still needed in clinical practice to help diagnose the prognosis of different stages and subtypes of endometrial cancer. This article studies the role of high-throughput measurement technology in cancer molecular typing and provides a theoretical reference for subsequent related research.

## 2. Related Work

After high-throughput genomic biotechnology was proposed, many scholars have developed some methods to predict the sensitivity of anticancer drugs. NCI adjusted the screening method, the screening subject changed from in vivo mice to human cell lines cultured in vitro, and NCI-60 and some other projects used cell lines as an intermediary to connect the genome and drug sensitivity. Some genomic markers related to drug response were obtained from it, and they were applied to clinical treatment with success. The literature [6] researched that kinase inhibitors such as verofenib have clinical therapeutic effects on BRAF and EGFR mutations. Researchers utilised gene expression profile information from the literature [7]. Gene expression in drug-resistant leukaemia cells was investigated by the literature [8], which revealed an association between the expression of illness recurrence-associated genes. The literature [9] suggested a co-expression extrapolation method to forecast the sensitivity of anticancer medicines and conduct research on particular kinds of cancer by analysing the specificity of gene expression between sensitive and drug-resistant cells. The literature [10] observes the drug's response to the cell by means of methylation marker nucleotide sequence. There is a wealth of scientific material in the literature [11], including gene mutations, copy number variations, and frequent cancer forms. It gives significant data support for evaluating anticancer drug responses in cell lines and considerably aids anticancer drug response prediction. The literature [12] suggested an elastic network regression model to predict the stability of medications based on gene expression, gene mutation, and copy number variation to investigate the association between anticancer drug sensitivity and the genome. The literature [13] fully considered the drug's chemical properties and genomic information and established a machine learning model to predict the response of cancer cell lines to drug treatment. The Bayesian matrix factorization model of the kernel approach uses drug sensitivity and genetic data to estimate missing values [14]. Using exome and transcriptome sequencing data to predict cancer cell line treatment response, the literature [15] developed a large-scale mechanical model parameterized computational framework. A model comparable to the recommendation system (CaDRReS) was suggested in the literature [16] and is based on the learning projection of cell lines and medicines to predict the response of anticancer treatments to unknown cell lines, thus accessing the possible drug genome space.

Those mutations that occur in cancer driver genes and play an important role in tumor production are called driver mutations [17]. Correspondingly, in the process of tumor production, mutations that do not promote the process of cancer are called passenger mutations [18]. This further explains that the occurrence of cancer is due to the accumulation of gene mutations, rather than a single gene mutation. Since different cancer types correspond to different driver mutations, finding the corresponding driver mutations for each type of cancer is helpful for prescribing the right medicine in medical treatment and launching targeted treatment. Although passenger mutation also plays a certain role in the development of cancer, its inducing effect on cancer is minimal compared to driver mutation. Therefore, effectively digging out the driving mutations in the mutation data is of great significance for future targeted therapy of cancer [19].

## 3. High-Throughput Sequencing Technology and Driving Gene Set Screening Model Based on Multiobjective Optimization

- Matrix *A* is an mxn matrix, as illustrated in Figure 1, to better understand the algorithm model. The columns and rows represent the number of different patient samples, whereas the rows represent the number of different genes. Black blocks correspond to 1, indicating that the gene is mutated, and white blocks correspond to 0, indicating that the gene is not altered, in the matrix. To put it another way, if we know how big the driving gene set is, we can convert the search into a search for a *K*-column submatrix that meets specific criteria in the mutation matrix Using the Dendrix algorithm, the study objective is the identification of driving pathway gene sets in somatic mutation data. The method is based on the drive path's two primary characteristics:
- High coverage: for the gene set in a certain cancer driving pathway, it is necessary to cover as many patient samples as possible. In other words, in the same type of cancer, most patients have at least one mutant gene that belongs to this driver gene set. As shown in Figure 1, when *K* = 2, in the two submatrices *B* and *C*, it is obvious that the submatrix *C* covers more patient samples than the submatrix *B*. However, the final screened gene set is matrix *B*. This is because while considering high coverage, another channel characteristic must be considered
- High exclusivity: each patient has a single mutation in the gene set that is the cause of the disease. This explains why matrix *B* is chosen in the end, despite matrix *C*'s superior coverage. As can be seen in Figure 1, matrix *D* contains a lot of overlapping patient samples, while matrix *B* has a decent exclusivity despite having somewhat poorer coverage.

Due to the actual mutation data, it is difficult to have the same result as the matrix *D* shown in Figure 1 when *K* = 3 and at the same time satisfy the coverage of all patients without a single patient sample with overlapping coverage. Therefore, a maximum weight submatrix model is constructed in the Dendrix algorithm. The model defines a weight function to weigh the relationship between coverage and exclusivity, which guarantees that both characteristics are satisfied at the same time. The specific form of the weight function is as follows.

(1) $$\begin{array}{c} W\left(M\right)=\left|\Gamma \left(M\right)\right|-\omega \left(M\right)=2\left|\Gamma \left(M\right)\right|-\underset{j\in M}{\sum }\left|\Gamma \left(j\right)\right|, \end{array}$$

Among them, *M*_*m*×*K*_ is the *K* column maximum weight submatrix obtained from the mutation matrix *A*, Γ(*j*) = {*i* : *A*_*ij*_ = 1} represents the sample set of all patients when gene *j* is mutated, and |Γ(*M*)| = *U*_*j*∈*M*_Γ(*j*) is a measure of coverage, indicating the patient samples corresponding to all gene mutations in the *M* matrix Set, *ω*(*M*) = *U*_*j*∈*M*_|Γ(*j*)| − Γ(*M*) is a measure of exclusivity, indicating the number of repeated coverage of all samples in the *M* matrix.

People often anticipate cheap prices and high quality from the goods they buy. However, high-quality goods need more expensive manufacturing, which drives up the price. Multiobjective optimization is all about finding a good balance between several goals to maximize the overall goal function. This is the key. The Pareto optimum solution is found at this point of equilibrium. The mathematical form of the multiobjective optimization problem is as follows:

(2) $$\begin{array}{c} f\left(X\right)=\left(f_{1}\left(X\right),f_{2}\left(X\right),\cdots ,f_{n}\left(X\right)\right). \end{array}$$

Among them, *f*(*X*) is the total objective function containing *n* single objectives, *X* is the decision vector, and S is a set of constraint conditions used to limit the parameter settings in each objective function.

Because the maximum weight submatrix model is based on two characteristics of the pathway gene set, high coverage and high exclusivity, a method for driving gene set search is proposed. The maximum weight submatrix we looked at is obviously a multiobjective optimization issue. The two objectives of coverage and exclusivity are weighted using the greatest weight objective function. Therefore, on the basis of the Dendrix algorithm, Dr. Zhao Junfei of the Chinese Academy of Sciences proposed the idea of using linear integer programming to solve the problem of solving the maximum weight submatrix model, and transformed the maximum weight submatrix model into the following mathematical form of the linear programming model. In the following, they are all referred to as BLP models.

(3) $$\begin{array}{c} \max F\left(x,y\right)=\max\left(f_{c}\left(x,y\right),f_{e}\left(x,y\right)\right)=\overset{m}{\underset{i=1}{\sum }}x_{i}-\left(\overset{m}{\underset{j=1}{\sum }}\left(y_{i}\overset{m}{\underset{i=1}{\sum }}a_{ij}\right)-\overset{m}{\underset{i=1}{\sum }}x_{i}\right)=2\overset{m}{\underset{i=1}{\sum }}x_{i}-\overset{m}{\underset{j=1}{\sum }}\left(y_{i}\overset{m}{\underset{i=1}{\sum }}a_{ij}\right),\\ \text{s}.\text{t}.\left\{\begin{array}{c} \overset{n}{\underset{i=1}{\sum }}a_{ij}y_{j}\geq x_{i},i=1,\cdots ,m;j=1,\cdots ,n,\\ \overset{n}{\underset{j=1}{\sum }}y_{j}=K,\\ x_{i},y_{i}\in \left[0,1\right]. \end{array}\right. \end{array}$$

Among them, *f*_*c*_(*x*, *y*) = ∑_*i*=1_^*m*^*x*_*i*_ represents the objective function of measuring coverage, and *f*_*e*_(*x*, *y*) = ∑_*j*=1_^*m*^(*y*_*j*_∑_*i*=1_^*m*^*a*_*ij*_) − ∑_*i*=1_^*m*^*x*_*i*_ represents the objective function of measuring exclusiveness. Among them, *K* represents the number of genes in the *M* matrix, *x*_*i*_ = {0, 1] represents whether the gene in the *i*-th patient sample falls into the *M* matrix has a mutation, the mutation is 1, otherwise it is recorded as 0, *y*_*i*_ = {0, 1] represents whether the *j*-th gene falls into *M* ‘matrix. If it falls in, it is 1, otherwise it is recorded as 0. *x* and *y* are vectors composed of *x*_*i*_ and *y*_*j*_, respectively.

The BLP model can accurately calculate the solution set of the maximum weight submatrix problem by adopting the idea of branching and defining, which not only solves the NP problem, but also solves the problem that Dendrix algorithm is easy to fall into local optimality. Moreover, this model is much faster than Dendrix when dealing with sparsely structured mutation matrices, which is very suitable for the analysis of large-scale mutation data.

Gene mutation heterogeneity is one of the characteristics of tumors is heterogeneity between tumors and heterogeneity within tumors.

These three gene variables and their impact on the frequency of gene mutations were studied using numerical experiments reported in this paper.  Figure 2 depicts the end outcome. The tumour genome atlas database (TCGA) provided the gene covariate data, and the details of the data are provided in this paper. There is evidence that the covariate data can be used in other cancer experimental studies.

According to Figure 2, we can analyze the correlation between the three gene covariates and the gene mutation frequency and find from the cross-correlation graph between the three covariates that there is a relationship between each gene covariate. Relevant studies have proved that the replication time of different regions of the genome is closely related to the level of gene expression and the state of chromatin. Genes with a highly spiral chromosome and a greater degree of gene expression replicate sooner. Genes with a long replication time, on the other hand, have a loose chromosomal state and little or no gene expression. As a result, the gene replication time is chosen as the most relevant covariate determining the frequency of gene mutations and integrated into the algorithm in this study to minimise the complexity of the method.

Gene replication time is identified as the intrinsic covariate that has the most effect on the frequency of gene mutation in this study. It is also examined quantitatively to see how the three different gene covariates interact with one another.

This article presents a novel search methodology for driver gene sets based on the effect of gene replication time. The following are the stages involved in creating the model:

1. The algorithm constructs the mutation matrix *A*_*m*×*n*_. *m* is the sample number of an independent patient, and *n* is the gene name. As shown in Figure 3, *A*_*ij*_ = 1 indicates that the *j*-th gene of the *i*-th patient has a mutation

(2) The algorithm defines the maximum weight submatrix function based on the influence of gene covariates:

(4) $$\begin{array}{c} W\left(M\right)=\left|\Gamma \left(M\right)\right|-\omega \left(M\right)=2\left|\Gamma \left(M\right)\right|-\underset{j\in M}{\sum }\left|\Gamma \left(j\right)\right|. \end{array}$$

The above model can also be transformed into a binary linear programming problem for solution:

(5) $$\begin{array}{c} \text{s}.\text{t}.\left\{\begin{array}{c} \overset{n}{\underset{i=1}{\sum }}a_{ij}y_{j}\geq x_{i},i=1,\cdots ,m;j=1,\cdots ,n,\\ \overset{n}{\underset{j=1}{\sum }}y_{j}=K,\\ x_{i},y_{i}\in \left[0,1\right]. \end{array}\right. \end{array}$$

Among them, *K* represents the number of genes in the *M* matrix, and *x*_*i*_ = {0, 1] represents whether the gene in the *i*-th patient sample falls into the *M* matrix has a mutation. If it has a sudden change, it is 1, otherwise it is recorded as 0. *y*_*i*_ = {0, 1] represents whether the *j*-th gene falls into the *M* matrix. If it falls in, then it is 1, otherwise it is recorded as 0. *x* and *y* are vectors composed of *x*_*i*_ and *y*_*j*_, respectively, and *λ*_*i*_ is the covariate weight value of the *j*-th gene.

This article considers the use of heuristic optimization algorithms. Multiobjective optimization problem solving methods are mainly divided into traditional optimization algorithms and intelligent optimization algorithms.

1. Traditional optimization algorithm

The classic traditional optimization algorithms include linear weighting method, norm weighting method and evolution method. The essence of this kind of method is to adopt the weighted idea, by transforming the multiobjective optimization problem into a single-objective optimization problem, and use the single-objective optimization method to solve it at the same time. This type of algorithm also has some shortcomings, specifically as follows:

- The unit quantification of various objective functions may be inconsistent and it is difficult for comparison to force weighting together
- The weighting coefficient is uncertainly chosen
- The progress of any individual goal in the overall optimization process is difficult to manage since it is the weighted sum of numerous single objective functions

This results in an extremely complex topology of the total optimization objective function, since choice variables, i.e., weighted coefficients, constrain each other.

(2) Algorithm for intelligent optimization

Genetic Algorithm (GA), Particle Swarm Optimization (PSO), Ant Colony Optimization (ACO), and other evolutionary algorithms are examples of intelligent optimization methods (EA). By replicating reproduction, competition, mutation, and selection in the process of biological evolution, this kind of algorithm creates a highly applicable global probability optimization search approach. The evolutionary algorithm uses the three phases of selection, crossover, and mutation to find the best solution to the optimization issue, similar to how biological evolution works. The evolutionary algorithm's basic principle is to start with a set of randomly generated populations and repeatedly perform selection, crossover, and mutation operations on them over multiple iterations, thereby improving the fitness of the population's individuals and gradually approaching the Pareto optimal solution set.

The ant colony method is a probabilistic search technique that is often used to address combinatorial optimization issues. This approach has solved travel salesman difficulties, graph colouring problems, communication networks, integrated circuit design, and vehicle scheduling challenges. Compared with other optimization algorithms, ant colony algorithm has the following three advantages:

1. The algorithm adopts the information positive feedback mechanism, which makes the convergence speed in the search iteration process continue to accelerate, and finally quickly approximates the optimal solution
2. Pheromone is time-sensitive, and its concentration will decrease over time, forming a negative feedback mechanism. This can effectively avoid the accumulation of too many pheromones on certain paths, leading to premature algorithms, that is, falling into local optimality

The algorithm adopts a distributed operation strategy in the iterative process, and all ants in the ant colony perform parallel operation at the same time, which greatly improves the operation efficiency of the algorithm.

Ant colony algorithm's most classic application scenario is to solve the Travelling Salesman Problem (TSP) problem. In this section, the process steps of ant colony algorithm will be briefly explained in combination with this problem.

The traveling salesman problem is that in *n* cities, each city can only pass through once, and it is required to find the shortest path that will eventually return to the starting point. Obviously, the TSP problem is also a combinatorial optimization problem. The problem can also be described in the following mathematical form.

(6) $$\begin{array}{c} \min D=\overset{n-1}{\underset{i=1}{\sum }}d\left(i,i+1\right)+d\left(n,i\right). \end{array}$$

Among them, *D* represents the optimal path, and *d*(*i*, *j*)(*i*, *j* = 1, 2, ⋯, *n*) represents the distance between city *i* and city *j*.

When using the ant colony algorithm to solve the TSP problem, there are *n* cities and *m* ants in the ant colony. In an iteration process, each ant decides the path to choose according to the probability of each path. The calculation formula for selection probability is as follows:

(7) $$\begin{array}{c} p_{i,j}^{k}\left(t\right)=\left\{\begin{array}{c} \frac{\tau_{ij}^{\alpha }\left(t\right)\eta_{ij}^{\beta }\left(t\right)}{\sum_{s\notin \text{Tabu}\left(\text{k}\right)}\tau_{\text{is}}^{\alpha }\left(t\right)\eta_{\text{is}}^{\beta }\left(t\right)},\;j\notin \text{Tabu}\left(\text{k}\right),\\ 0,\;j\notin \text{Tabu}\left(\text{k}\right), \end{array}\right. \end{array}$$

In the formula, *τ*_*ij*_(*t*) represents the pheromone concentration on the path from city *i* to city *j* at time *t*. At the initial time of the iteration, it is set to a constant c. *η*_*ij*_(*t*) represents the heuristic function. The calculation method is *η*_*ij*_(*t*) = 1/*d*(*i*, *j*), which reflects the degree of expectation that *i* transfers to city *j*. *α* is the information heuristic factor, used to regulate the importance of pheromone, *β* is the expected heuristic factor, used to regulate the importance of the heuristic function. tabu(k) is a taboo table, which means the list of cities that the *k*-th ant has traveled in an iteration, avoiding the path that has been traveled. When all the cities are included in the taboo table of ant *k*, this iteration of ant *k* is over. When every ant in the ant colony has completed this iteration. It is necessary to update the density of information on the route between each city. The adjustment formula is as follows:

(8) $$\begin{array}{c} \tau_{ij}=\left(1-\rho \right)\tau_{ij}+\Delta \tau_{ij},\\ \Delta \tau_{ij}=\overset{m}{\underset{k=1}{\sum }}\Delta \tau_{ij}^{k}. \end{array}$$

*ρ* is the pheromone volatilization coefficient, *ρ* ∈ (0, 1), *τ*_*ij*_ represents the pheromone intensity at a certain moment, and Δ*τ*_*ij*_^*k*^ represents the pheromone released by the *k*-th ant on the path from city *i* to city *j* during this iteration.

The steps of the entire ant colony algorithm can also be explained with the following Figure 4.

The 0-1 knapsack problem was proposed by Merkel and Hellman in 1978.The description of the problem is: Given a weight-bearing backpack and *n* items, the weight of each item *i* is *w*_*i*_ and the value is *v*_*i*_.Each item has only one piece and cannot be divided, and the item is either packed into a backpack or not packed into a backpack. In this case, how to choose the combination of items to maximize the total value of the backpack without being overweight can also be described by the following mathematical formula:

(9) $$\begin{array}{c} \begin{array}{c} \max f\left(x_{1},x_{2},\cdots ,x_{n}\right)=\overset{n}{\underset{i=1}{\sum }}v_{i}x_{i}\\ \text{s}.\text{t}.\overset{n}{\underset{i=1}{\sum }}w_{i}x_{i}\leq \text{Weight},\;x_{i}\in \left\{0,1\right\}\left(i=1,2,\cdots ,n\right). \end{array} \end{array}$$

To compare with the search model for driving gene sets in this article, the weight value is calculated according to the defined weight objective function for each combination of gene sets when *K* and *A* are given, and finally the gene set with a greater weight value is selected as the driving path analysis Candidate gene sets. Genes are either chosen into the candidate gene set or not based on the mutation frequency they exhibit when exposed to the covariate. It is clear that the issue is a classic 0-1 knapsack one. That is, selecting the item that optimises the overall worth of the backpack becomes a challenge when the backpack's load-bearing capability is restricted.

In the search for cell signaling pathways, each gene has only one and cannot be divided. Therefore, we use the weight of the backpack to control the number of genes *K* in the gene set. Since we are concerned about the number of genes in the gene set, the quality *w*_*i*_ of each gene is set to 1, and the value *v*_*i*_ of each gene corresponds to the number of gene mutations under the influence of the covariate. At the same time, we describe whether genes fall into our limited-size gene set as whether an item is loaded into a limited-weight backpack.

When more and more pheromone accumulates on a gene, the greater the probability that this gene will eventually fall into the resulting gene set. Each ant in the ant colony decides the gene to be selected according to the probability of gene selection in one iteration. The following formula represents the selection probability of the *k*-th ant for gene *g*:

(10) $$\begin{array}{c} p_{g}^{k}\left(t\right)=\left\{\begin{array}{c} \frac{\tau_{g}^{\alpha }\left(t\right)\eta_{g}^{\beta }\left(t\right)}{\sum_{s\notin \text{Tabu}\left(\text{k}\right)}\tau_{s}^{\alpha }\left(t\right)\eta_{s}^{\beta }\left(t\right)},j\in \text{Tabu}\left(\text{k}\right),\\ 0,g\in \text{Tabu}\left(\text{k}\right). \end{array}\right. \end{array}$$

Tabu(k) is a taboo table, a history record table of genes selected by the *k*-th ant in one iteration. The function is to avoid repeated selection of genes that have fallen into the gene set. *τ*_*g*_(*t*) is the pheromone intensity of gene *g* at time *t*, and *η*_*g*_(*t*) is the heuristic function. When solving the knapsack problem, we usually set *η*_*g*_(*t*) = *c*_*g*_/*w*_*g*_. *c*_*g*_ is the “value” of gene *g*, *w*_*g*_ is the “quality” of gene *g*, and *η*_*g*_ represents the “unit value” of gene *g*. *α* is the information heuristic factor, which controls the importance of the pheromone, and *β* is the expected heuristic factor, which controls the importance of the heuristic function.

After each ant selects a gene, it needs to judge whether the quality of the backpack at this time exceeds the load-bearing value, that is, whether the number of selected genes exceeds the set gene set size *K*. When each ant in the ant colony has completed all the selections in an iteration, the pheromone accumulated on each gene must be adjusted once. The adjustment formula is:

(11) $$\begin{array}{c} \left\{\begin{array}{c} \tau_{g}\left(t+n\right)=\left(1-\rho \right)\tau_{g}\left(t\right)+\Delta \tau_{g}\left(t\right),\\ \Delta \tau_{g}\left(t\right)=\overset{m}{\underset{k=1}{\sum }}\Delta \tau_{g}^{k}\left(t\right). \end{array}\right. \end{array}$$

Among them, *ρ* is the pheromone volatilization coefficient, *ρ* ∈ (0, 1); *τ*_*g*_(*t* + *n*) represents the pheromone intensity of gene *g* at time *t* + *n*, and Δ*τ*_*g*_^*k*^(*t*) represents the pheromone released by the *k*-th ant on gene *g* during this iteration. The calculation formula is:

(12) $$\begin{array}{c} \Delta \tau_{g}^{k}\left(t\right)=\left\{\begin{array}{c} c_{g}\times \frac{Q}{c^{k}},\;g\in g^{k},\\ 0,\;g\notin g^{k}. \end{array}\right. \end{array}$$

In the formula, *Q* represents the information intensity, which is a constant, and *g*^*k*^ represents the list of genes selected by the *k*-th ant in this iteration, and is the “total value” of the genes selected by the *k*-th ant. This article adjusts the parameters through experiments, and finally sets the experimental parameters to *α* = 2, *β* = 5, *p* = 0.5, *Q* = 100, and ant colony size *m* = 30.

When all the iterative processes are completed, calculate the value of each ant's backpack, and the corresponding gene in the backpack with the greatest value is the gene set we selected.  Table 1 is the pseudocode of the ACDP algorithm, which can be implemented in various programming languages.

## 4. Research on Cancer Molecular Typing Based on High-Throughput Sequencing Technology

Many high-throughput sequencing data sets are widely used. However, identifying cancer driver genes requires the use of excellent databases that satisfy practical application requirements. Somatic mutation data sets, network and route data sets, and protein interaction network data sets are three types of data sets that may be classified based on their intended use (PPIs).

This cost may be decreased indefinitely as technology and application development progresses. This new technique can break through many of the current roadblocks in the study of cancer illness. This high-throughput technique makes it possible to study huge numbers of malignant tumours at a cheap cost. This opens the door to a more in-depth look at cancer from many perspectives, including the genome, transcriptome, proteome, and others (Figure 5).

Currently, the more popular data sets are: a: Somatic Mutations Data Collection (1) COSMIC (the catalogue of somatic mutations in cancer) is now the most used and largest somatic mutation database. The COSMIC database records the somatic mutation information of various types of human malignant tumors. The database has the following characteristics: (1) It keeps detailed records of mutation locations, including information such as the exact mutation content, cancer kinds associated with it, literature associated with it, and sample names, among other things. As a result, it includes complete statistical information for a particular mutant gene as well as information on cancer tissue and cancer cell lines at various stages of cancer. Additionally, information on the fusion gene is provided. As a result, researchers can better understand the role of somatic mutations in cancer. (2) In 2006, the American Cancer Institute and the American Institutes of Health collaborated to establish TCGA (The Cancer Genome Atlas). Its goal is to uncover all oncogene and tumor suppressor gene mutations throughout the carcinogenesis process and perfect the genome sequencing of more than 50 malignancies or cancer subtypes. This database is the biggest cancer gene information resource presently available, offering extensive assistance for the research of cancer molecular pathways. The TCGA project has completed research on more than 36 cancer types, and its database has steadily grown to become the most significant source of original data in cancer research. (3) Cancer3D is a very user-friendly database. In the kinase research community, 3D structural information plays a critical role in discovering driver mutations. Cancer3D is a database that examines somatic missense mutations based on the 3D structure of proteins. With the use of this annotated database, scientists can figure out how protein 3D structure affects somatic mutations. b: Set of information on the pathways. Kyoto Encyclopedia of Genes and Genomes (KEGG) is an online resource for learning about biological systems' intricate workings. In order to investigate pathogenic mutations and somatic mutations that have a functional effect in cancer, it intends to encompass all cell signalling pathways. A useful feature of the database is that it offers users with input genes for enrichment analysis, making it easier to discover novel cancer-related signal pathways. The database (2) The Reactome database is a tool for studying biological processes in general. It aims to gather articles related to various reactions and biological pathways in the human body, which are often written, reviewed and reviewed by experts. The database provides an effective data source and related e-books for channel research. (3) PID (Pathway Interaction Database) was founded by the National Cancer Institute (NCI) and Nature Publishing Group. Users can query specific information about cell signal pathways and cell signal regulation processes known to the human body by molecular names or metabolic process names. (C) Protein interaction network data set; (1) BioGRID (Biological General Repository for Interaction Datasets) was created in 2003 and is a database that stores data about interactions between proteins and genes. The data is mainly obtained by mining the literature on protein interactions. (3) IntAct is a free and open source molecular interaction database, derived from the European Institute of Bioinformatics. Most of the data comes from literature mining and other related molecular interaction databases. Moreover, a good search process and graphical search results are also the highlights of this database.

There are five types of cancer driver mutation research techniques used nowadays. Methods based on mutation frequency include the following characteristics: When using the conventional frequency approach, researchers look for genes with mutation rates that are substantially greater than the sample's background rate using statistical methods. This technique has inherent limitations as a result of tumour heterogeneity and the impact of other variables. Some better solutions have been presented to overcome this issue. To find driving mutation genes, the OncoddriveCLUST method, for example, constructs a background model based on silent mutations and groups mutations with substantial mutation propensity in particular protein areas. In actual applications, this approach has yielded positive outcomes. (2) A approach based on the effect of functional factors. Researchers must immediately establish an efficient approach to sequence the driving mutation genes due to high-throughput sequencing technologies' vast quantity of mutation data. Researchers now have tools to swiftly measure mutations' functional impact because of the advent of computational approaches. Theoretically, these methods might aid researchers in identifying prospective genes for future scientific study. The SIFT (Sorting Intolerant from Tolerant) method, for example, is a common biological study tool that predicts missense mutations based on protein sequence homology. (3) Genome-structure-based approaches. Technology like nuclear magnetic resonance, X-rays, and high-quality 3D protein structure sequencing back up this approach. According to the research, mutations in key nodes in the signalling system have been linked to disease therapy and therapeutic targets. Considering the signal pathway topology, protein structure, and other information will definitely enhance the algorithmic efficiency while looking for potential driver mutations. According to these studies, the technique of enhancing signal channels via topological structure has shown promising outcomes in biological trials. (4) Pathway and network analysis method. Cells are a complex and dynamic network composed of a variety of molecular structures. Gene mutations may affect or remove a node in the network, and even affect the biological characteristics of the node, thereby further leading to changes in the network structure. Therefore, the method based on the path and the network has high applicability. (5) Data integration method. This is a method for researchers to systematically study the mechanism of driving mutations and cancer by including a variety of omics data. It is often necessary to establish a mathematical model to integrate a variety of omics data. The integrated model proposed in this paper has the characteristics of this method.

## 5. Conclusion

The patient's physical state and clinical reaction symptoms are usually used as the foundation for screening medications from various compounds based on experience to reach a fair diagnosis in the conventional clinical treatment technique. According to research, there are considerable variances in cancer's sensitivity to chemotherapeutic treatments, and tumors in various organs and systems have distinct features. Due to the differences in disease kinds, even though it is the same tissue and portion, the degree of sensitivity to the medicine will be quite varied. The same form of cancer may react to the same therapy in various ways. As a consequence, various drugs should be utilised even while treating the same kind of cancer. The diagnosis and treatment approaches used in the past are no longer enough for today's cancer treatment needs. Due to the rapid rise of modern biotechnology and big data analysis technology, many experimental investigations have acquired a substantial quantity of biomedical data, and biomedical information has been continually upgraded. Consequently, modern humans must address the biological problem of determining how to mine biological data for meaning and laws. Precision medicine is defined as medicine based on the pathological traits of patients, such as biological data such as cells, genes, and proteins, as well as the characteristics of the sickness, to build a treatment plan for the appropriate patient. Precision medicine encourages the study of personalized genetic data and the development of focused medical treatments for individuals based on their biological data. This article investigates the function of high-throughput measurement technology in molecular cancer typing in order to encourage the growth of the medical sector better. It also serves as a theoretical reference for future related research.

## Figures and Tables

**Figure 1:** Mutation matrix.

**Figure 2:** The correlation between gene covariates and gene mutation frequency.

**Figure 3:** Mutation matrix.

**Figure 4:** Flow chart of the ant colony algorithm.

**Figure 5:** Canceromics research strategy.

**Table 1:** Interpretation of some variables in the pseudocode.

Variable	Explanation
*m*	The number of ants in the colony
maxstep	The maximum number of iterations
maxvalue_*t*	The maximum value of the gene set during the *t*-th iteration
bestplan	In all iterations, the gene number corresponding to the most valuable gene set
maxvalue	In all iterations, the maximum value of the gene set selected by the ant colony
gene_set	The corresponding number of the gene set in the mutation matrix

## Data Availability

The data used to support the findings of this study are included within the article.
